The article "Differentiation of Small Gastrointestinal Stromal Tumor and Gastric Leiomyoma with Contrast-Enhanced CT" was published in 2023. Journal: J Healthc Eng.

# Differentiation of Small Gastrointestinal Stromal Tumor and Gastric Leiomyoma with Contrast-Enhanced CT

**DOI:** 10.1155/2023/6423617

**Published:** 2023-02-08

**Authors:** Mingyan Yan, Yubao Liu, Honglian You, Yanbo Zhao, Jun Jin, Jing Wang

**Affiliations:** ^1^Department of Radiology, Shenzhen Qianhai Shekou Free Trade Zone Hospital, Shenzhen 518000, China; ^2^Imaging Center, Shenzhen Hospital of Southern Medical University, Shenzhen 518100, China

## Abstract

**Objective:**

The value of multiphase contrast-enhanced CT in differentiating gastrointestinal stromal tumors (GISTs) and gastric leiomyomas (GLMs) which were ≤3 cm was evaluated using machine learning.

**Methods:**

A retrospective analysis was conducted on 45 cases of small gastric wall submucosal tumors (including 22 GISTs and 23 GLMs) with pathologically confirmed diameter ≤3 cm and completed multiphase CT-enhanced scan images. The CT features including tumor location, maximum diameter, shape, margins, growth pattern, plain/enhanced CT value, cystic degeneration, calcification, ulcer, progressive reinforcement, perilesional lymph nodes, and the CT value ratio of the tumor to the aorta at the same level in the enhanced phase III scan of the two groups were evaluated. Tumor location and maximum diameter were automatically evaluated by machine learning.

**Results:**

The GISTs and GLMs with a diameter ≤3 cm showed clear margins, uniform density on plain scan CT, and progressive homogeneous enhancement. The age of the GISTs is greater than that of the GLMs group. The plain scan CT value of the GISTs group was lower than that in the GLMs group. In the GISTs group, the lesions were mostly located in the fundus (68.18%), showing a mixed growth pattern (54.55%), and in the GLMs group, most lesions were located in the cardia (47.82%), showing an intraluminal growth pattern (95.65%). The abovementioned differences were statistically significant.

**Conclusions:**

Contrast-enhanced CT has limited value in differentiating small GISTs from GLMs, which are ≤3 cm. Older age (>49.0 years), a low plain CT value (<42.5 Hu), mixed growth inside and outside the cavity, and noncardiac location tended to be the criteria for the diagnosis of small GISTs of the gastric wall.

## 1. Introduction

Gastrointestinal stromal tumors (GISTs) and gastric leiomyomas (GLMs) are two common tumors derived from gastrointestinal mesenchymal tissue. GISTs are Cajal cells originating from the muscularis propria of the gastrointestinal wall and have malignant potential [1], while GLMs are benign tumors originating from the smooth muscle tissue of the gastrointestinal wall [2]. GIST lesions vary in size, and their imaging manifestations are diverse, with round, quasi-round, or irregular shapes. Necrotic cystic degeneration, hemorrhage, and calcification may occur in the lesions. Enhanced scanning shows uniform or uneven enhancement, most of which are obvious, and vascular-like enhancement can be seen in some arterial phases, while necrosis and cystic degeneration are not significantly enhanced. GLMs mostly occur in the stomach. In addition to direct invasion and distant metastasis suggesting malignancy, irregular or lobulated tumors, uneven enhancement, central necrosis, ulceration, and uneven thickening of the adjacent intestinal wall suggest a high possibility of LMs. Submucosal tumors of the stomach wall with diameter ≤3 cm in the GISTs are GISTs with a decreasing diameter, and the value of multiphase CT enhancement in the identification of gastric wall GISTs and GLMs is limited. Among them, only older age, a lower plain CT value, mixed growth inside and outside the cavity, and occurrence in the gastric fundus are more inclined to the diagnosis of small GISTs in the gastric wall.

Previous studies on the differential diagnosis of the two tumors in imaging are not lacking. With the increasing widespread clinical application of digestive endoscopy, more and more small gastric wall submucosal tumors have been discovered and attracted attention [3]. As the tumor diameter decreases, its imaging features are incharacteristic, which makes differential diagnosis more difficult, and preoperative differentiation between small GISTs and GLMs is important for treatment selection. In this study, multiphase enhanced CT images of gastric wall submucosal tumors with a diameter of ≤3 cm were retrospectively analyzed to explore their imaging manifestations and the basis for differential diagnosis.

## 2. Materials and Methods

### 2.1. Research Object

A total of 78 cases of pathologically diagnosed gastric wall submucosal tumors were treated by endoscopic ultrasonic-guidedfine-needle puncture or endoscopic/surgical resection from June 2018 to June 2021. Among them, there were 35 cases of GISTs, 31 cases of GLMs, 5 cases of gastric schwannoma, 4 cases of ectopic pancreas, 1 case of gastric polyp, 1 case of gastric cancer, and 1 case of glomus tumor. GISTs and GLMs with a diameter of ≤3 cm were included in this study, and cases without preoperative CT enhancement or poor image quality were excluded. Finally, 45 cases were included, including 22 cases of GISTs and 23 cases of GLMs.

### 2.2. Inspection Method

All examinations were performed with a 256-slice multislice CT scanner (Revolution CT, GE, USA). Before the CT examination, the patient fasted for 4–6 hours, and 500–1000 mL of water was taken orally 10 minutes before the scan (to fully dilate the stomach and duodenum). Scanning parameters were as follows: tube voltage 120 kV, Smart mA technology, speed 0.5 s, pitch 1.375, layer thickness 5 mm. The reconstruction layer thickness is 1.25 mm. The patient underwent breathing training. After the plain scan, a high-pressure syringe was used to inject a nonionic iodinated contrast agent (iohexol, 300 mgI/mL, 1.2 ml/kg) through the antecubital vein at a flow rate of 2.5–3.5 ml/s, and the scan was triggered by the smart tracking technology. The abdominal aorta layer was monitored; the trigger threshold was 120 Hu. The breathing command was deep inhalation and then breath-holding, and multiphase CT-enhanced scanning was performed in the arterial phase (5.9 s), the portal venous phase (20 s), and the delayed phase (120 s) by automatically triggering the enhanced scanning. The tube was flushed with 30 ml of normal saline after the injection.

### 2.3. Research Method

The blind method is used. The CT images were retrospectively analyzed by two imaging diagnosticians (with working years of 15  and 7 years, respectively), and the differences were resolved through consultation. The contents of analysis include tumor location, maximum diameter, shape, margins, growth pattern (intraluminal or mixed type, this group of cases is small, and there is no single extraluminal growth case), plain scan and enhanced CT values at each stage (select the largest level of the lesion, the area of uniform density, the area of interest 2∼4 mm^2^, the average CT value), the presence or absence of cystic calcification, enhancement mode (the difference between the CT value of the most obvious part of the lesion and the weakest part of the enhancement is less than 10 Hu defined as uniform enhancement, greater than or equal to 10 Hu for heterogeneous enhancement), lymph nodes around the lesion (shorter diameter greater than 5 mm), and the ratio of the three-phase enhancement of the lesion to the CT value of the aorta at the same level (R-A, R-V, R-D). When measuring aortic CT values, the ROI was enlarged as much as possible, and the average value was taken. Tumor location and maximum diameters were automatically evaluated using machine learning by GE software (GE Milwaukee, USA).

### 2.4. Statistical Analysis

SPSS 26.0 statistical software was used. Measurement data (age, maximum diameter of tumor, plain/enhanced CT value, and R-A/V/D) between two groups were compared by a *t*-test or Mann–Whitney *U* test. Data were expressed as mean ± standard deviation ($\bar{x}\pm s$) or median (upper and lower interquartile range: M (P25, P75)). A chi-square test or adjusted chi-square test was used to compare count data (sex, tumor location, morphological margin, growth pattern, presence or absence of cystic calcification, and enhancement pattern) between the two groups. The receiver operating characteristic (ROC) curve was used to determine the best cutoff value (the sum of specificity and sensitivity was the highest) to distinguish GISTs from GLMs, Youden value = sensitivity−(1−specificity). *P* < 0.05 was statistically significant.

## 3. Results

### 3.1. Comparison of General Clinical Data and CT Features

A total of 45 patients were included in this study, including 20 males and 25 females, aged from 27 to 68 years old, with an average age of (51.00 ± 11.10) years, and lesion sizes ranging from 0.8 to 3.0 cm. Among them, there were 22 cases of the small GISTs in the gastric wall (pathology showed extremely low risk in 15 cases, low risk in 6 cases, and medium risk in 1 case) and 23 cases of the small GLMs in the gastric wall. The average age, maximum size of the tumor, plain CT value, multistage enhanced CT value, the ratio of the three-phase enhancement of the lesion to the CT value of the aorta at the same level, tumor location, morphology, tumor margin, growth mode, cystic change, calcification, enhancement mode, and adjacent enlarged lymph nodes of the two groups are shown in Table 1. The median age of the GISTs is greater than the median age of the GLMs group (*P* < 0.05). The plain CT value of GISTs was lower than that of the GLMs group (*P* < 0.05). 15/22 (68.18%) of the small GISTs in the gastric wall are located in the fundus of the stomach (Figure 1), and the 11/23 (47.83%) of small GLMs in the stomach wall are located in the cardia (Figure 2). The small GISTs in the stomach wall with mixed growth in the intraluminal/extraluminal are about 12/22 (54.55%) (Figure 1), whereas the GLMs are mainly with intraluminal growth (Figure 2) and are about 22/23 (95.65%) (*P* < 0.05).

### 3.2. Receiver Operating Characteristic (ROC) Curve

The ROC curve showed that when patients were older than 49.50 years old, the area under the curve, sensitivity, and specificity for diagnosing GISTs were 0.836, 86.4%, and 73.9%, respectively (Figure 3). When the unenhanced CT value was greater than 42.5 Hu, the area under the curve, sensitivity, and specificity for diagnosing GLMs were 0.777, 69.6%, and 77.3%, respectively (Figure 4).

## 4. Discussion

With the wide application of digestive endoscopy, the detection of gastric subepithelial lesions has greatly increased, especially the small GISTs in the gastric wall with a diameter of ≤3 cm. Due to its inert biological characteristics, some scholars suggest that it should be classified as a special type or even a benign tumor to be distinguished. So what is the imaging performance and identification basis of such small GISTs and small GLMs? Is there any change compared with conventional lesions reported in the literature?

This study showed that the average age of the small GISTs group was greater than that of the GLMs group, which was consistent with the results of previous studies [4]. The ROC curve showed that when the patient was older than 49.50 years old, the area under the curve, sensitivity, and specificity of GISTs were 0.836, 86.4%, and 73.9%, respectively, indicating that older age at onset can also be used as the basis for the identification of gastric small GISTs and small GLMs.

Choi et al. studied that the gastric corpus is the predisposing site of GISTs in the gastric wall [5], and the risk of GISTs increases as the GISTs move down in the gastric cavity compared with the gastric cardia [6]. In this study, the small GISTs were mostly located in the gastric fundus, and 95.45% were in the low-risk or very low-risk group. Cardia or involvement of the gastroesophageal junction is a significant feature of GLMs [5, 7]. In this study, about 47.82% of small GLMs occurred in the cardia. Therefore, the occurrence of lesions in the gastric fundus or the cardia becomes one of the important basis for the identification of gastric wall small GISTs and small GLMs.

The plain CT value of the GISTs group was lower than that of the GLMs group. The ROC curve showed that when the unenhanced CT value was greater than 42.5 Hu, the area under the curve, sensitivity, and specificity for diagnosing GLMs were 0.777, 69.6%, and 77.3%, respectively. In the past, the imaging characteristics of GISTs have rarely paid attention to the CT value of a plain scan, and more attention has been paid to whether the density of the lesion is uniform and whether there is cystic necrosis and hemorrhage. These signs suggest an increased risk of malignancy and become the main basis for distinguishing GISTs from other benign tumors of the gastric wall. In our study, the small lesions had clear margins and uniform enhancement on both plain and enhanced scans, indicating the characteristics of low or very low malignancy. The lower CT value of a plain scan has become one of the bases for diagnosing small GISTs.

In terms of tumor growth patterns, the lesions in the GISTs group showed mixed growth, and the lesions in the GLMs group grew into the cavity, which may be due to the different histological sites of the two tumors. Endoscopic ultrasonography shows that gastric wall GISTs mostly occur in the fourth layer of the gastric wall, namely, the muscularis propria, so they can grow both inside and outside the cavity [6]. GLMs mostly originate from the third layer, the muscularis mucosae, so they grow toward the mucosal surface with less growth resistance and protrude into the lumen, which is consistent with the results of previous studies [7–9], indicating that the histological location and growth pattern of small GISTs are similar to conventional lesions.

In previous studies, in GISTs tumors with a diameter of 2–5 cm or larger, the cystic degeneration, lobulation, inhomogeneous enhancement, and surface ulcers suggested a higher risk of GISTs and became the main basis for differentiating them from GLMs [5, 10]. However, the abovementioned signs in this study of small lesions did not have any distinguishing value. Both lesions showed progressive enhancement with a clear margin and uniformity, showing the imaging manifestations of benign spindle cell-derived tumors. The disadvantage of this study is that the sample size is small, and we look forward to expanding the sample size in the future and further exploring its diagnostic and differential diagnosis characteristics through radiomics methods.

## Figures and Tables

**Figure 1:** A 63-year-old man with small GISTs in the stomach wall. ① Plain CT scan revealing an oval mixed growth of soft tissue mass in the fundus of the stomach, smooth with clear margin and a maximum diameter of 2.1 cm. The CT value of plain CT scan was 32 Hu, showing mixed growth in the intraluminal/extraluminal. ②–④ Enhancement scanning of the arterial phase, venous phase, and delayed phase, resulting in uniform progressive enhancement of the mass.

**Figure 2:** A 37-year-old man with small GLMs in the gastric wall. ① Plain CT scan showing a soft tissue mass growing in an oval cavity from the cardia, smooth with clear edge and a maximum diameter of 2.7 cm. The CT value was 38 Hu and the mass grew inside the cavity. ②–④ Enhancement scanning of the arterial phase, venous phase, and delayed phase, respectively, resulting in homogeneous enhancement of the mass.

**Figure 3:** ROC curves of age-diagnosed GISTs.

**Figure 4:** ROC curve for the diagnosis of GLMs by plain CT values.

**Table 1:** Comparison of general clinical data and CT features between small gastric GISTs and GLMs (*n* (%)).

	GISTs group (22 cases)	GLMs group (23 cases)	Statistical	*P* value
Gender			1.779^①^	0.182
Male	12 (54.54)	8 (34.78)		
Female	10 (45.46)	15 (65.22)		
Average age (years)	60.50 (51.00, 64.25)	47.00 (37.00, 54.00)	−3.863^④^	<0.001^∗^
Tumor location			13.276^①^	0.001^∗^
Cardia	2 (9.09)	11 (47.83)		
Fundus of stomach	15 (68.18)	4 (17.39)		
Gastric body	5 (22.73)	8 (34.78)		
Tumor shape			0.987^②^	1.000
Smooth	22 (100)	22 (95.65)		
Lobular	0 (0)	1 (4.35)		
Tumor margin			2.222^②^	0.243
Clear	20 (90.91)	17 (73.91)		
Verge	2 (9.09)	6 (26.09)		
Growth mode			13.792^①^	<0.001^∗^
Intraluminal	10 (45.45)	22 (95.65)		
Mixed	12 (54.55)	1 (4.35)		
Cystic change			0.301^②^	0.489
Yes	1 (4.76)	0 (0)		
No	21 (95.24)	23 (100)		
Calcification			0.001^②^	1.000
Yes	1 (4.76)	1 (4.35)		
No	21 (95.24)	22 (95.65)		
Enhancement mode			0.178^②^	1.000
Homogeneous	20 (90.91)	20 (86.96)		
Inhomogeneous	2 (9.09)	3 (13.04)		
Progressive enhancement			0.650^①^	0.420
Yes	15 (68.18)	13 (56.52)		
No	7 (31.82)	10 (43.48)		
Adjacent enlarged lymph nodes			2.001^②^	0.489
Yes	0 (0)	2 (8.70)		
No	22 (100)	21 (91.30)		
Tumor maximum diameter (cm)	1.80 (1.40, 2.33)	1.30 (1.10, 1.90)	−1.707^④^	0.088
Plain CT value (Hu)	37.32 ± 7.82	46.48 ± 8.63	−3.727^③^	0.001^∗^
CT value of phase A (Hu)	57.50 ± 12.31	59.65 ± 8.93	−0.674^③^	0.504
R-A	0.19 (0.15, 0.21)	0.18 (0.17, 0.21)	−0.352^④^	0.725
CT value of phase V (Hu)	69.86 ± 11.74	67.43 ± 9.63	0.760^③^	0.451
R–V	0.49 (0.45, 0.55)	0.44 (0.42, 0.52)	−1.953^④^	0.051
CT value of phase D (Hu)	73.23 ± 11.95	73.43 ± 10.05	−0.063^③^	0.950
R-D	0.71 ± 0.10	0.68 ± 0.09	1.140^③^	0.261

*Note.* ① represents the chi-square test, ② represents the correction chi-square test, ③ represents the *T* test, ④ represents the Mann−Whitney *U* test; ^∗^indicates a statistical difference.

## Data Availability

The data used to support the findings of this study are available from the corresponding author upon reasonable request.
